# Analysis of Clinical Manifestations, Imaging Features, and Gene Mutation Characteristics of 6 Children with Cystic Fibrosis in China

This article has been retracted.

**DOI:** 10.1155/2021/7254391

**Published:** 2021-11-02

**Authors:** Yajuan Chu, Jinfeng Shuai, Kunling Huang, Jianhua Liu, Wenshan Lv, Baochi Li

**Affiliations:** Department of Respiratory Medicine, Hebei Children's Hospital, Shijiazhuang, Hebei 050031, China

## Abstract

**Objective:**

To explore the clinical manifestations, imaging features, and gene mutation characteristics of 6 children with cystic fibrosis (CF) so as to improve the understanding and diagnosis awareness of CF in children and reduce the missed diagnosis and misdiagnosis.

**Methods:**

The clinical manifestations, imaging, and gene mutation data of six children with CF were collected and retrospectively analyzed.

**Results:**

Among the 6 cases of CF, there were 4 males and 2 females. Among the 6 children with CF, 5 cases presented with recurrent respiratory tract infection. Etiology suggested 3 cases of *Pseudomonas aeruginosa* and 2 cases of *Staphylococcus aureus*. 3 cases had pancreatic exocrine dysfunction, manifested as diarrhea and aliphatic diarrhea, of which 1 case had high lipase in blood examination, and pancreatic ultrasound showed rough and enhanced pancreatic echo, considering pancreatic cystic fibrosis. 2 cases of CF combined with pseudo-Bartter syndrome (PBS); 1 case involved only the biliary tract and started with cholestasis without other systemic involvement. In 2 cases of sweat test, sweat chloride ions were all >60 mmol/L. 3 cases underwent fiberoptic bronchoscopy, and a large number of sticky secretions were visible under the bronchoscopy. CT of the chest revealed thickening of the bronchial wall (3 cases), bronchiectasis (1 case), atelectasis (1 case), and thin bronchial lumen (2 cases). 1 patient was found to have small airway lesions and mosaic perfusion during follow-up. All 6 children with CF underwent genetic testing. A total of 12 CF transmembrane conductance regulator (CFTR) gene mutations were found, of which 4 mutations were not reported in the literature.

**Conclusion:**

CF is a disease caused by CFTR mutation. The incidence of this disease in China is low, and the clinical manifestations have great differences. The main symptoms are respiratory symptoms. Some children have gastrointestinal symptoms and/or PBS, and some children only show a single systemic lesion.

## 1. Introduction

Cystic fibrosis (CF) is an autosomal recessive genetic disease, and it is the deficiency of CF transmembrane conductance regulator (CFTR) protein function caused by the mutation of CFTR gene [1]. CF can cause a large amount of mucus to block the exocrine glands of the body, which can affect multiple systems such as respiration, digestion, and reproduction. The clinical manifestations of CF include chronic cough, cough up a lot of sputum, recurrent pulmonary infection, steatosis, growth retardation, and male infertility [2, 3]. The CFTR gene is located in the first band of the third region of the long arm of chromosome 7 and contains 27 exons. So far, more than 2,000 genetic variations have been found to affect the function of CFTR protein through different mechanisms [4]. CF is one of the common hereditary diseases in the Caucasian population, and the incidence rate is 1/1800 to 1/25000 [5]. In the Asian population, the incidence of CF is low, and the incidence varies from region to region. In Japan, 104 cases of CF that occurred in Japan from 1951 to 1993 are summarized, and the incidence rate of CF in Japan is considered to be about 1/350000 [6]. In China, the incidence of CF is low, and no epidemiological statistics are available. The previous incidence of CF in China is likely to be underestimated due to insufficient understanding and imperfect detection technology. However, in recent years, with the improvement of clinicians' understanding of CF and the development of gene detection technology, the diagnosis rate of CF increases year by year. If clinicians have insufficient knowledge of CF and imperfect detection methods, this may cause delay in diagnosis and treatment. Therefore, in order to understand the basic manifestations of CF, we collected the clinical manifestations, imaging features, and gene mutation characteristics data of 6 children with diagnosed CF and conducted a retrospective analysis, in order to accurately and early diagnose CF, which is of great significance for individualized treatment of children.

## 2. Methods

### 2.1. General Information

6 children with CF who were hospitalized in Hebei Children's Hospital from July 2018 to April 2021 were selected as the research subjects.

#### 2.1.1. Diagnostic Criteria for CF

The diagnosis of CF requires a combination of unique clinical manifestations, sweat tests, and/or CFTR dysfunction. CF diagnostic procedure: for patients with one or more clinically characteristic phenotypes, such as chronic and recurrent sinus and lung disease, malnutrition, digestive tract disease, male genitourinary system malformations (such as absent vas deferens), or a family history of CF, sweat chloride detection was performed. If the secondary sweat chloride ion ≥60 mmol/L or one time sweat chloride ion ≥40 mmol/L +2 pathogenic mutations of CFTR, CF could be diagnosed.

#### 2.1.2. Diagnostic Criteria for Pancreatic Cystic Fibrosis

Children with CF have clinical manifestations of impaired pancreas. It is mainly the absorption disorder of fat, protein, and saccharides caused by pancreatic exocrine dysfunction, which can present with diarrhea and weight loss, and in severe cases, it can cause such symptoms as fatty diarrhea, malnutrition, and growth retardation. Imaging examinations revealed signs of damaged pancreas, such as plump pancreas, nonuniform echo of pancreatic parenchyma, pancreatic steatosis, pancreatic fibrosis, pancreatic dilatation, pancreatic atrophy, and cystic degeneration of the pancreas.

#### 2.1.3. Diagnostic Criteria for Pseudo-Bartter Syndrome (PBS)

When hypokalemia, hyponatremia, hypochloremia, and alkalosis occur in some children, their clinical manifestations were similar to Batter syndrome.

### 2.2. Research Methods

The basic information, clinical manifestations, laboratory tests, imaging characteristics, gene mutation characteristics, and treatment of 6 hospitalized children diagnosed with CF were analyzed retrospectively through the hospital electronic medical record system. Low-dose chest CT was performed in all children with CF. The chest CT manifestations included bronchiectasis, bronchial wall thickening, mucus plug, lung consolidation, atelectasis, mosaic perfusion and tree bud sign, and other signs, and the distribution was evaluated. With the informed consent of the parents, 2 mL peripheral blood samples was collected from all children with CF and the 27 exons and blank sequences of CFTR gene were amplified by polymerase chain reaction (PCR). Exon capture was performed using Agilent SureSelect method, and high-throughput sequencing was performed using Illumina sequencing platform. After the sequencing data were matched and analyzed by software, mutation screening and explanation were performed using Ingenuity online software system. The candidate mutations were verified by Sanger sequencing.

## 3. Results

### 3.1. Basic Information

Among the 6 cases of CF, there were 4 males and 2 females. The initial onset age of symptoms was 2.25 ± 2.51 months, and the definitive diagnosis age was (9.83 ± 7.57) months. All 6 cases were sporadic; the parents of all the children were married not close relatives, and there were no patients with similar diseases in the family.

### 3.2. Clinical Manifestations and Laboratory Test Results

Among the 6 children with CF, 5 cases presented with recurrent respiratory tract infection. Etiology suggested 3 cases of *Pseudomonas aeruginosa* and 2 cases of *Staphylococcus aureus*. 3 cases had pancreatic exocrine dysfunction, manifested as diarrhea and aliphatic diarrhea, of which, 1 case had high lipase in blood examination, and pancreatic ultrasound showed rough and enhanced pancreatic echo, considering pancreatic cystic fibrosis. 2 cases of CF combined with PBS; 1 case involved only the biliary tract and started with cholestasis without other systemic involvement. In 2 cases of sweat test, sweat chloride ions were all >60 mmol/L, as shown in Table 1.

  Case 1: male, with a respiratory tract infection at the age of 2 months, manifested as cough and wheeze, viscous sputum with diarrhea and aliphatic diarrhea, excessive sweating, sweat crystals on his skin, and pulmonary function suggestive of moderate obstructive ventilatory dysfunction. Auxiliary examinations—blood routine tests: white blood cells (9.8–17.6) *∗* 10^9^/L, neutrophil percentage 29.6%–45.9%, hemoglobin 98–112 g/L, platelet (240–308)*∗*10^9^/L, and C-reactive protein 5.78–14.36 mg/L; liver functions: alanine aminotransferase 80 U/L, aspartate aminotransferase 83 U/L; no abnormality was found in blood amylase; blood lipase 119.4 U/L, increased; a plurality of times of alveolar lavage fluid culture for *Pseudomonas aeruginosa*; sweat test result: chloride 140 mmol/L.
  Case 2: male, with a respiratory tract infection at the age of 7 months, manifested as cough, expectoration, and wheezing without diarrhea was investigated for liver function abnormalities; pulmonary function tests showed moderate-to-severe obstructive ventilatory dysfunction. Auxiliary examinations—blood routine tests: white blood cells 11.1*∗*10^9^/L, neutrophil percentage 63.8%, hemoglobin 128 g/L, platelet 431*∗*10^9^/L, and C-reactive protein <0.5 mg/L; stool routine: liposome 27–33/HPF, amyloid granule 1–5/HPF; liver function: alanine aminotransferase 78 U/L, aspartate aminotransferase 57 U/L; electrolytes, calcium, and glucose, renal function, and myocardial enzymes were almost normal. The alveolar lavage fluid was cultured for *Pseudomonas aeruginosa*; sweat test result: chloride 110 mmol/L.
  Case 3: female, onset of respiratory infection at 3 months of age, accompanied by diarrhea, steatorrhea, growth retardation, and abnormal liver function. Auxiliary examination: blood routine examination—white blood cells 11.2*∗*10^9^/L, neutrophil percentage 34.4%, hemoglobin 97 g/L, platelet 202*∗*10^9^/L, C-reactive protein 6.89 mg/L; stool routine: fat globule: 30–45/HPF; erythrocyte sedimentation rate: 46 mm/h; liver functions: 69 U/L alanine aminotransferase, 99 U/L aspartate aminotransferase, and 157 U/L gamma-glutamyl transpeptidase; blood amylase: 18 U/L. The bronchoalveolar lavage fluid was cultured for *Staphylococcus aureus*.
  Case 4: male, meconium excretion was delayed after birth; pneumonia and diarrhea occurred in the neonatal period. At the age of seven months, he was hospitalized because of poor spirit for more than one month, drowsiness for half a month, and cough for four days. During this period, diarrhea still occurred and the stool was yellow. The fat globules were routinely visible through stool examination, and the lung function indicated moderate obstructive ventilatory dysfunction. Auxiliary examination: blood routine examination—white blood cells 7.1*∗*10^9^/L, neutrophil percentage 48.9%, lymphocyte percentage 43.8%, hemoglobin 117 g/L, platelet 346*∗*10^9^/L, and C- reactive protein 1.99 mg/L; blood electrolytes: K^+^2.04 mmol/L, Na^+^124.7 mmol/L, Cl^−^54.6 mmol/L; blood gas analysis: PH7.631, increased. Sputum culture showed *Staphylococcus aureus*. The child was suffering from hypokalemia, low sodium, low chlorine, and alkalosis; the initial diagnosis did not exclude Batter syndrome, and further examination of urinary potassium, urinary sodium, and urinary chlorine were normal.
  Case 5: female, with yellow sclera staining of her skin on the 3rd day after birth. The jaundice improved after symptomatic treatment and then became worse again. She was hospitalized for 54 days after birth; liver function tests: total bilirubin 188.9 *μ*m mol/L, direct bilirubin 154.4 *μ*m mol/L, total bile acid 127.1 *μ*m mol/L, gamma-glutamyl transpeptidase 55 U/L, alanine aminotransferase 110 U/L, and aspartate aminotransferase 135 U/L. Auxiliary examination: blood routine examination—white blood cells 7.61*∗*10^9^/L, neutrophil percentage 18.9%, lymphocyte percentage 69.7%, hemoglobin 104 g/L, platelet 373*∗*10^9^/L, and C-reactive protein 1.1 mg/L.
  Case 6: male, with a respiratory tract infection at the age of 1 years, manifested as nasal congestion, cough, fever, and runny nose, with pulmonary function suggestive of a mild obstructive ventilatory dysfunction prior to relaxation, and electrolyte metabolism disorders (low sodium, low potassium, and low chlorine) combined with metabolic alkalosis during the second hospitalization, considering a combination of PBS. Auxiliary examination: blood routine examination—white blood cells 6.1*∗*10^9^/L, neutrophil percentage 41.5%, lymphocyte percentage 44.0%, hemoglobin 131 g/L, platelet 234*∗*10^9^/L, and C-reactive protein 15.41 mg/L. Bacterial culture of bronchoalveolar lavage fluid was *Pseudomonas aeruginosa*.

### 3.3. Image Features

3 cases underwent fiberoptic bronchoscopy, and a large number of sticky secretions were visible under the bronchoscopy. CT of the chest revealed thickening of the bronchial wall (3 cases), bronchiectasis (1 case), atelectasis (1 case), and thin bronchial lumen (2 cases). 1 patient was found to have small airway lesions and mosaic perfusion during follow-up (Figures 1–9), as shown in Table 2.

  Case 1: pancreas ultrasound: coarse enhancement of pancreatic echo; CT of the chest showed inflammation in both lungs, with uneven light transmittance, thickened tracheal wall, partial bronchiectasis and bronchiectasis; bronchoscopy revealed a large amount of yellow viscous purulent discharge with cloudy lavage fluid. During the follow-up, the child's small airway lesions and mosaic-like perfusion was found in the child.
  Case 2: chest CT scan showed patchy shadows, thickening of the bronchial wall, bronchial stenosis, and bronchiectasis; bronchoscopy revealed a large amount of viscous secretion attachment; observation under the transmission electron microscope of pathology of bronchial mucosa showed that cilia were locally visible, with irregular cilia, short and sparse cilia, and occasionally syndesmophyte cilia that were mixed and distributed with microvilli, and a large number of cilia with 9 + 2 microtubule structure abnormalities could be seen, which were manifested as falling off of cilia outer membrane, loss of internal and external power arm, radiolysis, and preservation of central microtubule, consistent with the ultrastructural pathological changes of primary ciliary immobility syndrome.
  Case 3: chest CT showed consolidation, atelectasis, uneven opacity, and normal lung function; fiberoptic bronchoscopy revealed a large amount of viscous secretions and bronchoalveolar lavage fluid culture of methicillin-resistant *Staphylococcus aureus*; sinus CT : inflammation of left maxillary sinus with slightly thickened mucosa of right maxillary sinus and bilateral ethmoid sinus.
  Case 4: pancreas ultrasound showed homogeneous solid echo; sputum culture for *Staphylococcus aureus*; pulmonary function suggests moderate obstructive ventilatory dysfunction. On chest CT, multiple patchy high-density shadows were observed in both lungs, with unclear boundary with pleura, thickening of right costal pleura, patency of trachea and bronchus, no migration of mediastinum, and no effusion in both thoracic cavities.
  Case 5: cholestatic liver disease was considered because of abdominal ultrasound suggesting an unfilled gallbladder, increased and enhanced echogenicity of the liver parenchyma, and a thin (0.5 mm) diameter of the extrahepatic bile duct.
  Case 6: the thorax was symmetrical, and no abnormality was found in the soft tissue of the chest wall. The trachea and left and right main bronchi were patent, and patchy shadows could be seen in the left lung and the lower lobe of the right lung. The bronchial walls in the lower lobes of both lungs were slightly thick, the bronchi in the lower lobe of the right lung were slightly widened, and the bilateral hilars were not large.

### 3.4. Gene Mutation Characteristics

All 6 children with CF underwent genetic testing. A total of 12 CFTR gene mutations were found, of which 4 mutations were not reported in the literature (Figures 10–15), as shown in Table 3.

  Case 1: CFTR had two heterozygous mutations, 577G > A was carried by the father and 2547C > A was carried by the mother. The child was diagnosed with CF and pancreatic cystic fibrosis.
  Case 2: exon 23 heterozygous mutation c.3796_3797dupGA in our child detected by NGS sequencing and confirmed by Sanger sequencing to be from the mother; an exon 15 heterozygous deletion was detected by MLPA, which was verified by QPCR to be from the father, and neither of the two CFTR variants was reported in the literature. Although electron microscopy of the bronchial mucosa revealed primary ciliary immobility, CF was finally diagnosed in combination with the child's clinical presentation, sweat test, and CFTR gene variation.
  Case 3: CFTR had two heterozygous mutations, 1159_1160delTT was carried by the father and 2328dupA was carried by the mother. Diagnosis of CF based on clinical manifestations and genetic results.
  Case 4: CFTR with a homozygous mutation of 2909G > A combined with clinical presentation, genetic test results, electrolyte disturbance, and metabolic alkalosis led to the final diagnosis of CF combined with PBS.
  Case 5: CFTR had two heterozygous mutations: 374T > C was carried by the mother and 2950G > A was carried by the father. Combined with the clinical manifestations and CFTR gene mutation, CF was finally diagnosed definitively.
  Case 6: CFTR had three heterozygous mutations: 3484C > T was carried by the mother, 2909G > A was carried by the father, and 3717 + 45G > A was carried by the mother. Combined with the clinical manifestations, gene test results, electrolyte disorders, and metabolic alkalosis, PBS was considered to be combined.

### 3.5. Treatment

The treatment of CF is mainly aimed at clinical manifestations and complications. The treatment of pulmonary diseases includes active control of infection, strengthening management of respiratory tract infection and anti-inflammatory treatment, and giving treatments such as bronchoalveolar lavage, cefoperazone and sulbactam for anti-infection, and oral pancreatin replacement. Nutritional therapy includes supplementation of trypsin, fat-soluble vitamins, minerals, and high-energy foods; other treatments include correction of electrolyte imbalance, liver protection and enzyme reduction, and oral administration of ursodeoxycholic acid. All 6 children with CF received systematic treatment and received follow-up treatment in the outpatient department on a regular basis to give symptomatic treatment.

## 4. Discussion

CF is a hereditary exocrine gland disease that affects multiple systems of the body and affects the life span of children, and it is a disease caused by CFTR gene mutation [7]. The disease can lead to decreased secretion of Cl^−^ and water by epithelial cells of exocrine gland duct, resulting in increased content of sodium chloride in exocrine fluid, viscous and unsmooth secretion drainage, and obstruction of lumen of respiratory tract, pancreas, sweat gland, biliary tract, and other organs, with consequent corresponding clinical manifestations. The clinical manifestations of CF vary greatly, mainly including respiratory symptoms, manifested as repeated respiratory tract infections, accompanied by atelectasis and bronchiectasis, and followed by pulmonary function decline and respiratory failure. Respiratory symptoms are the most important cause of death for CF [8]. Foreign studies have reported that the clinical manifestations of CF in Caucasians are often acute or recurrent respiratory diseases (43.6%), developmental delay (24.9%), chronic diarrhea/fatty diarrhea/malnutrition (20.4%), and meconium intestinal obstruction (14.2%), while the manifestations of chronic sinusitis and nasal polyps are relatively rare (4.4%), and about 10.2% of children have a positive family history [9]. Among children with CF in China, the most common pathogen is *Pseudomonas aeruginosa*, followed by *Staphylococcus aureus*, *Klebsiella pneumoniae*, and other pathogens. In this study, among the 6 children with CF, 5 cases showed repeated respiratory tract infections, manifested as cough, sputum, and wheeze. The etiology suggested *Pseudomonas aeruginosa* in 3 cases and *Staphylococcus aureus* in 2 cases.

At present, it is clinically known that CF is a fatal disease in infancy and childhood. With the continuous development of medical technology in recent years, clinicians have an increased understanding of CF, which improves the survival rate of children with CF. However, studies have shown that progressive lung disease still accounts for more than 95% of deaths in children with CF [10]. For children with CF, morphological changes often occur in infancy and are usually not reflected in the lung function measurement before the age of 4. Therefore, it is necessary for clinicians to monitor the lung condition of children with CF as soon as possible [11]. The main features of chest CT are bronchiectasis, thickening of the bronchial tube wall, or mucus impaction in the expanded bronchus, which is related to the increase and thickening of mucus and poor dissolution. Stiglbauer's team [12] reported that through chest CT report, it could be known that CF could present with bronchiectasis, thickening of bronchial wall, mucus plugs, cystic degeneration or lung abscess, lung bulla, air retention, and atelectasis or lung consolidation. The thickening of bronchial wall, bronchiectasis, and mucus plugs were relatively common, especially in the upper lobes of both lungs, but no significant difference was observed between the two lungs. In six cases of this group, chest CT showed bronchial wall thickening (3 cases), bronchiectasis (1 case), atelectasis (1 case), and bronchiectasis (2 cases). The follow-up visit of one case revealed a small airway lesion with mosaic perfusion, which was the manifestation of small airway involvement, and the upper lobes of both lungs were more common. This result is basically consistent with the research results of imaging characteristics of CF patients reported by Yang et al. [13]. Sinusitis is another manifestation of CF involving the upper respiratory tract. The sinus CT of Case 3 in this study showed inflammation of left maxillary sinus with slightly thickened mucosa of right maxillary sinus and bilateral ethmoid sinus, and unaeration of bilateral frontal sinuses and sphenoid sinuses, which proved high viscosity and consistency with the pathogenesis of CF.

In Caucasians, children with CF may involve multiple abdominal organs, and when pancreas is involved, it will present with pancreatic exocrine insufficiency, pancreatic steatosis, and pancreatic atrophy. When liver is involved, liver steatosis and cirrhosis will be manifested. When the biliary system and kidney are involved, the manifestations include gallstones, cholecystitis, bile duct stenosis, and kidney calculi [14]. We found that 4 cases had different degrees of obstructive ventilatory dysfunction, and 2 cases had normal ventilatory function. 3 cases underwent fiberoptic bronchoscopy, and a large number of sticky secretions were visible under the bronchoscopy. 3 cases of CF in this group had pancreatic exocrine dysfunction, which led to poor absorption, with the manifestations of diarrhea and aliphatic diarrhea. 1 case had high lipase in the blood examination, and pancreatic ultrasound showed rough and enhanced pancreatic echo, which diagnosed pancreatic cystic fibrosis. In addition, only 33% of children with CF have hepatobiliary disease in clinical practice, but its fatality rate ranks third, second only to lung infection and transplantation complications of CF. Cholestasis caused by CF is mainly due to the thick bile in the intrahepatic bile duct, increased acidic substances, and decreased formation of normal bile flow, with clinical manifestations of delayed meconium discharge or meconium intestinal obstruction, claylike stool, and even no gallbladder in the small gallbladder, which is easily confused with biliary atresia. Early life may not be accompanied by respiratory symptoms and other organ involvement, and biochemical characteristics mainly include direct bilirubin, glutamic acid transaminase, gamma-glutamyl transferase, and alkaline phosphatase increase. In this study, the cholestasis of the child in Case 5 was characterized by delayed meconium excretion and elevated direct bilirubin, without other system involvement. This child has no claylike stool, which is related to the child's young age. It is not ruled out that the color of the stool becomes lighter with age, and the clinician needs to follow up and pay attention to the child.

In infancy, children with CF mainly present with repeated respiratory tract infections, fatty diarrhea, and growth retardation, and 12%–18.8% of them present with low potassium, low sodium, low chlorine, and metabolic alkalosis as the initial or main manifestations, but without renal tubulopathy, which is known as PBS. The reason for PBS is that the sweat glands failed to effectively recover sodium and chloride ions due to the mutation of CFTR gene, and the body lost a large amount of water and electrolyte with sweat, thus activating the renin-angiotensin-aldosterone system and increasing the discharge of potassium ions, resulting in hypokalemia [15]. In addition, bicarbonate is accumulated in the body by increased compensatory absorption of bicarbonate and decreased glomerular filtration rate, eventually leading to electrolyte disorders and alkalosis. PBS can cause convulsion, hypovolemia, arrhythmia, and severe cases can even lead to death. Risk factors for PBS include small infants, hot weather, fever, respiratory tract infection, vomiting, and diarrhea. The onset of hot weather with symptoms of respiratory tract infection and diarrhea prompted Case 4 and Case 6 of our group to incorporate PBS. In clinical work, if children suffer from hyponatremia, hypochlorohypokalemia, and metabolic alkalosis that cannot be explained by other diseases such as Batter syndrome, diuretic use, and pyloric obstruction, physicians should be alert to the possibility of PBS caused by CF.

Sweat detection is an important and accurate method for detecting CF. The chloride ion concentration in sweat of children with CF is usually higher than 60 mmol/L. Sweat test was performed on two children with CF in this group. The chloride ions in sweat of the children were all >60 mmol/L. However, sweat test is very strict with the operator's operation. Small errors in operation will cause errors in chloride ion concentration and affect the diagnosis. At present, only a few hospitals in China can implement sweat test. As a safe, fast, and easy method, gene detection also plays an important role in the diagnosis of CF. Diagnosis can be confirmed by genetic testing in children with atypical clinical presentations and/or negative (or threshold) sweat tests. CF is caused by a gene mutation on the long arm of chromosome 7. The gene-encoded product CFTR is a cAMP-regulated chloride channel protein located at the tip of exocrine gland epithelial cells. The gene mutation leads to abnormal synthesis and translation of this protein as well as loss of its function, reducing the permeability of epithelial cells of exocrine glands for chloride ions and increasing their absorption of sodium ions, causing intracellular hypertonic state with thick secretion, which can affect multiple organs and systems of the whole body. Until now, more than 2,000 mutations in the CFTR gene have been identified; however, only 10% of these mutations are common, and the majority are rare mutations with a low incidence. Some mutations are pathogenic. The most common gene mutation in Europe and North America is ∆F508, accounting for more than half [16]. However, the ∆F508 mutation is not common in Asians, and the ∆F508 mutation was not seen in the 6 children with CF in our study. In this study, all 6 children with CF underwent genetic testing. A total of 12 CFTR gene mutations were found, of which 4 mutations were not reported in the literature. Case 1 in this group was a typical CF case, presenting with the triad of chronic lung disease, pancreatic insufficiency, and elevated sweat chloride ion. Some mutations are sequence variations that do not cause CF; some of the mutations show only minor lesions or single systemic lesions, known as “CFTR-associated disease or CFTR-associated metabolic syndrome,” and Case 5 in this group involves only the biliary tract, starting with cholestasis and without other systemic manifestations. The 12 gene mutations in this study were not common mutations in Caucasians, so the gene mutation spectra of Chinese and Caucasians were quite different [17, 18].

It should be noted that CF should be distinguished from primary ciliary dyskinesia (PCD) in clinical practice [19]. PCD is an autosomal recessive genetic disease caused by abnormal ciliary movement. It is extremely rare and the main symptom of PCD is also repeated respiratory tract infection like CF, with clinical manifestations including cough, expectoration, bronchiectasis, sinusitis, otitis media, and infertility. The diagnosis of PCD requires the transmission electron microscope examination of ciliated epithelium of nasal or bronchial mucosa. Overseas studies have suggested that the electron microscope manifestation of PCD is mainly kinesin arm defect, accounting for about 70% to 80%. Microtubule deletion and disorder of microtubule arrangement are also the main electron microscope manifestations. In Case 2 of this group, repeated respiratory infections occurred in infancy, and chest CT indicated bronchiectasis in the upper lobe of the left lung. Under the electron microscope, a large number of cilia with 9 + 2 microtubule structure abnormalities were observed, manifesting as cilia outer membrane loss and missing of internal and external power arm. Without sweat test and gene detection results, PCD could be easily misdiagnosed. The sweat test of this child was >60 mmol/L, and the gene report indicated mutation of CFTR gene, one heterozygous mutation c.3796_3797dupGA, and one heterozygous deletion. The final diagnosis of CF was confirmed. The abnormal structure of cilia 9 + 2 microtubules in this child was considered to be related to repeated infections caused by CF. In addition, children with CF have an earlier age of onset, and most children start to get onset within 1 year of age, while children with PCD are more likely to have complications of otitis media. According to reports, CF is usually characterized by bronchiectasis in the upper lung field, which can be used as a reference basis for the differential diagnosis of PCD. Case 2 was onset at the age of 7 months without manifestations of otitis media, and bronchiectasis in the upper lobe of the left lung. The above characteristics can be used as the main points of identification.

The treatment of CF is multifaceted, mainly aiming at the clinical manifestations and complications, including infection control, removal of airway secretions, reduction of chronic inflammation, improvement of gastrointestinal function, and nutritional support. For patients with respiratory failure and pulmonary heart disease, lung transplantation may be considered. In addition, some progress has been made in gene targeted therapy. For example, ivacaftor was approved by the US FDA for marketing in 2012 and is mainly used for the treatment of specific G551D mutation. In 2019, the US FDA has processed applications for new drugs for the elexacaftor, tezacaftor, and ivacaftor triple therapy, which is used for treating CF patients with the age ≥12 years old, specifically, patients with one F508 del mutation and one minimal functional mutation, or patients with two F508 del mutations. Specific gene therapy for other mutations is also being studied. Active comprehensive treatment for children with CF can alleviate clinical symptoms, reduce mortality, and improve quality of life.

## 5. Conclusion

CF is a disease caused by CFTR mutation. The incidence of this disease in China is low, and the clinical manifestations have great differences. The main symptoms are respiratory symptoms. Some children have gastrointestinal symptoms and/or PBS, and some children only show a single systemic lesion. In China, the clinical manifestations and gene mutation sites of CF are different from those reported abroad, and some children with atypical clinical manifestations may be misdiagnosed or missed. In clinical work, we should improve the understanding of and attention to CF and assist in the diagnosis of suspected cases by genetic testing to accumulate clinical experience. With the development of molecular biology technology, gene detection will play a positive role in the early diagnosis, early treatment, and prognosis improvement of the disease. The shortcoming of this study is that CF usually involves multiple systems. However, in this study, the children with CF only involved the respiratory system, digestive system, or liver. At the same time, the number of cases in this study is small, and there are no manifestations of lung abscess, cystic degeneration, and bullae in this group of children. The association between Chinese genotype and clinical phenotype needs to be further explored in the light of the abundant cases.

## Figures and Tables

**Figure 1:** Chest CT manifestations of the child: inflammation in both lungs was visible, with uneven light transmittance, and the tracheal carina and right main bronchus, right upper lobe bronchus, and right middle lung bronchial lumen were thin.

**Figure 2:** Condition under fiberoptic bronchoscopy and alveolar lavage fluid: a large amount of yellow viscous purulent secretions were obstructed and attached to the bronchus, and the lavage fluid was turbid.

**Figure 3:** Inflammation of both lungs, bilateral bronchiolitis.

**Figure 4:** Chest CT examination: bilateral lung inflammation with small cyst cavity and initial stenosis of upper lobe bronchus in left lung were considered.

**Figure 5:** Fiberoptic bronchoscopy showed inflammation of the tracheobronchial intima with numerous cords and thrombi of secretion attached.

**Figure 6:** Chest CT examination: right lung inflammation and upper lobe segmental atelectasis of the right lung were considered.

**Figure 7:** What the sinus CT image showed: high-density shadow was seen in the left maxillary sinus, some mucous membranes of the right maxillary sinus and bilateral ethmoid sinus were slightly thickened, bilateral frontal sinus and sphenoid sinus were not gasified, the right maxillary sinus orifice was blocked, the left maxillary sinus orifice was unobstructed, the nasal septum was basically in the middle, and the bilateral middle turbinate and inferior turbinate were not large. No obvious abnormality is found in the soft tissue of the parietal and posterior wall of nasopharynx.

**Figure 8:** Chest CT examination: inflammation in both lungs with thickening of the right costal pleura.

**Figure 9:** Chest CT examination: inflammation in both lungs, slightly dilated bronchi in the lower lobe of the right lung.

**Figure 10:** Genetic analysis results.

**Figure 11:** Genetic analysis results.

**Figure 12:** Genetic analysis results.

**Figure 13:** Genetic analysis results.

**Figure 14:** Genetic analysis results.

**Figure 15:** Genetic analysis results.

**Table 1:** Clinical manifestations and laboratory test results of 6 children with CF.

Case	Gender	Age ofonset	Age of diagnosis	Main clinical manifestations	Pathogenicbacteria	Sweat chlorineconcentration (mmol/L)
Case 1	Male	2 months	5 months	Repeated respiratory tract infections, diarrhea, celiac disease, liver dysfunction, sweat crystals, moderate obstructive ventilatory dysfunction	*Pseudomonas aeruginosa*	140
Case 2	Male	7 months	2 years	Repeated respiratory tract infections, liver dysfunction, moderate-to-severe obstructive ventilatory dysfunction	*Pseudomonas aeruginosa*	110
Case 3	Female	3 months	5 months	Repeated respiratory tract infection, diarrhea, fatty diarrhea, abnormal liver function, normal lung function, growth retardation	*Staphylococcus aureus*	Not checked
Case 4	Male	12 days	9 months	Repeated respiratory tract infections, diarrhea, celiac disease, PBS, moderate obstructive ventilatory dysfunction	*Staphylococcus aureus*	Not checked
Case 5	Female	3 days	4 months	It begins with cholestasis, manifested as jaundice and abnormal liver function.	Not checked	Not checked
Case 6	Male	1 month	1 year	Repeated respiratory tract infections, combined with PBS, mild obstructive ventilatory dysfunction	*Pseudomonas aeruginosa*	Not checked

**Table 2:** Imaging features of 6 children with CF.

Case	Pulmonary imaging
Case 1	Patchy shadow, bronchial wall thickening, bronchiectasis, late mosaicism
Case 2	Patchy shadow, bronchial wall thickening, bronchiectasis, bronchiectasis
Case 3	Consolidation shadows, atelectasis, uneven opacity
Case 4	Patchy shadow
Case 5	Not checked
Case 6	Patchy shadow, bronchial wall thickening

**Table 3:** Gene mutation characteristics of 6 children with CF.

Case	Location	CFTR mutation site	Amino acid change	Variation type	Parentalgenotype	Genetic mode	Literature reporting
Case 1	Exon 5	c.577 G > A	p.E193X	Nonsense mutation	Father was a carrier	Compound heterozygosity	Reported
	Exon 15	c.2547C > A	p.Y849X	Nonsense mutation	Mother was carrier		

Case 2	Exon 23	c.3796_3797dupGA	p.I1267Kfs∗12	Frameshift mutation	Mother was carrier	Heterozygous mutation	Notreported
	Exon 15	Exon15 heterozygous deletion	—	Nonsense mutation	Father was a carrier	Heterozygous deficiency	

Case 3	Exon 9	c.1159_1160delTT	p.L387Nfs∗23	Frameshift mutation	Father was a carrier	Heterozygous mutation	Reported
	Exon 14	c.2328dupA	p.V777Sfs∗2	Frameshift mutation	Mother was carrier		Not reported

Case 4	Exon 18	c.2909G > A	p.G970D	Missense mutation	Parents were carriers	Homozygous mutation	Reported
Case 5	Exon 4	c.374T > C	p.I125T	Missense mutation	Mother was carrier	Heterozygous mutation	Reported
	Exon 18	c.2950G > A	p.D984N	Missense mutation	Father was a carrier		Not reported

Case 6	Exon 22	c.3484C > T	p.R1162X	Nonsense mutation	Mother was carrier	Heterozygous variation	Reported
	Exon 18	c.2909G > A	p.G970D	Missense mutation	Father was a carrier		
	Exon 22	c.3717 + 45G > A	Splicing	Splice mutation	Mother was carrier		

## Data Availability

The data used and/or analyzed during the current study are available from the corresponding author upon request.
